This article has been retracted.

# Application of Clavien–Dindo Classification System for Complications of Minimally Invasive Percutaneous Nephrolithotomy

**DOI:** 10.1155/2021/5361415

**Published:** 2021-12-15

**Authors:** Xiao-Jun Zhang, Zheng-Jie Zhu, Jun-Jie Wu

**Affiliations:** Department of Urology Surgery, The Affiliated Xiangshan Hospital of Wenzhou Medical University, Ningbo, Zhejiang Province 315700, China

## Abstract

**Objective:**

To investigate the clinical applications of the Clavien–Dindo classification system (CDCS) in the assessment of perioperative complications in minimally invasive percutaneous nephrolithotomy (MPCNL).

**Methods:**

Totally, 390 patients with renal stones in our hospital from March 2015 to March 2020 were included for this study and then were divided into observation group (complication group, 78 cases) and control group (noncomplication group, 312 cases) according to the incidence of perioperative complications in CDCS. Single factor analysis and multivariate logistic regression analysis were used to analyze the risk factors of the perioperative complications of MPCNL.

**Results:**

The total incidence of complication in the 390 cases with MPCNL was 20.00% (78 cases) according to CDCS, among which the incidence of complications at grades I, II, III, IV, and V was 6.92% (27 cases), 8.21% (32 cases), 2.82% (11 cases), 1.79% (7 cases), and 0.26% (1 case), respectively. The proportion of patients, that aged >60 years, complicated with comorbidities, sophisticated calculi, the preoperative albumin level (<35 g/L), the operation time (>180 minutes), intraoperative bleeding volume (>300 mL), and hospitalization time (>7 days) in the observation group was significantly higher than that in the control group ((75.64% vs. 61.86%, 38.46% vs. 24.36%, 83.33% vs. 69.55%, 83.33% vs. 69.55%, 70.51% vs. 30.76%, 53.85% vs. 36.54%, and 60.26% vs. 43.27%), all *P* < 0.05). Multivariate logistic regression analysis showed that gender, associated comorbidities, preoperative albumin level, calculus complexity, operation time, and intraoperative bleeding volume (>300 mL) were correlated with the occurrence of complications (*P* ≤ 0.001, 0.001, 0.001, 0.001, 0.003, and 0.001 respectively).

**Conclusion:**

The CDCS can give standard and more comparative criteria for the assessment of perioperative complications, which will provide reference data for reducing complications and ensuring safety profiles in these high-risk patients.

## 1. Introduction

Renal stones were one of the most common diseases in the urinary system, and it often occurs in the young and the middle-aged people; the morbidity was higher in males than females [1, 2]. Studies showed that, about 40% to 75% of patients with renal stones underwent different degrees of back pain, which is often taken as the primary clinical manifestation to visit doctors [3]. At the early stage, patients with small diameter stones and mild symptoms can alleviate the illness by drinking lots of water and physical exercises or other conservative treatments [4, 5]. However, with the influence of the patient's diets, environmental conditions, and other factors, the diameter of renal stones will be gradually enlarged in some people; consequently, the frequency and duration time of pain will increase, and hematuresis, hydronephrosis, or urinary tract obstruction would be found in some serious patients [6, 7]. When conservative treatment does not work for kidney stones, procedures such as transurethral ureteroscopic lithotripsy, percutaneous nephrolithotripsy, and laparoscopic ureterolithotripsy are often considered alternatives to conservative treatment. [8, 9].

Minimally invasive percutaneous nephrolithotomy (MPCNL) is a most common operation in urology, which was modified on the basis of percutaneous nephrolithotomy. MPCNL had the advantage of small trauma, high discharging rate, rapid recovering course, and so on. MPCNL was effective for renal stones, but the complications in the perioperative period did not receive enough attention compared with its clinical efficacy. And, the evaluation of complications was usually based on operator's experience, but lacked consistent criteria [10]. How to carry out quantitative evaluation and reduce the incidence of perioperative complications in MPCNL are becoming surgical hotspots. In order to investigate the criteria of standardized assessment and the risk factors of the complications of MPCNL, 390 patients with renal stones from March 2015 to March 2020 in our hospital were collected in the study, and the Clavien–Dindo classification system (CDCS) was adopted to analyze the perioperative complications.

## 2. Patients and Methods

### 2.1. Patient Data

Totally, 390 patients with renal stones who underwent MPCNL from March 2015 to March 2020 in our hospital were collected, including 254 males and 136 females; aged from 40 to 70 years; 274 urban patients and 116 rural patients; 156 patients with diabetes, hypertension, chronic bronchitis, or other general comorbidities, and 234 patients without comorbidity; and 255 patients with simple renal stones and 135 patients with complex renal stones [11] (including stone diameter >25 mm, horn-like or multiple renal stones, stones that are difficult to remove caused by abnormal anatomy, etc.).

### 2.2. Surgical Methods

Epidural anesthesia or general anesthesia with endotracheal intubation were performed in operation, these patients were performed or supervised by a single surgeon who had previous experience of MPCNL. All patients were placed in the lithotomy position with conventional sterilization of surgery area, and the surgical towels were placed. The 5 Fr or 6 Fr ureteral catheter was inserted to the target ureter directed by ureteroscopic vision. After uretheral catheter insertion, the patients were replaced in a prone position, and percutaneous access was achieved by fluoroscopic guidance using an 18–20-gauge needle. Patients were punctured under the direction of B ultrasound. Then, the ureteroscope (Richard wolf, Germany) was placed in the renal pelvis, and the holmium laser (Litho, Italy) was used to fragment renal stones. The stones were discharged under the pressure of the irrigation solution or were taken out with basket catheter. At the end of surgery, a nephrostomy tube was inserted and removed 1 week after surgery, the double *J* ureteral catheter was inserted into the renal pelvis and removed 1 month after surgery, and the operation time was calculated from the insertion of ureteral catheter to the placement of nephrostomy tube.

### 2.3. Classification Standards and Evaluation Methods

Perioperative complications were divided into grade I, II, III, IV, and V according to CDCS [12]. Grade I: the complications had mild impacts on patients' recovery, but there is no threat to the life of patients, and these antipyretics, analgesics, antiemetics, diuretics, and physical therapy were allowed to application. Grade II: on the basis of grade I, other kinds of drugs, blood infusion, or total intravenous nutrition were required. Grade III: surgery, endoscope, or radiotherapy were required, including grade IIIa and grade IIIb; grade IIIa did not require general anesthesia, which could be performed by surgical intervention directly; grade IIIb required to carry out general anesthesia. Grade IV: it includes grade IVa and grade IVb; the former one's complications having life threats to the patients, who showed single organ failure and needed ICU care, and the latter one manifested as multiple organ failure. Grade V: patients' death was caused by complications. The incidence of perioperative complications in patients was observed and recorded.

### 2.4. Statistical Analysis

The data were analyzed with SPSS22.0 statistical software; the measurement data was expressed as mean ± standard deviation (‾x±SD) and analyzed by the *t*-test; the numerical data were expressed as *n* (%) and analyzed by chi-square (*χ*^2^) test; the single factor analysis and multivariate logistic regression analysis were used to analyze the risk factors of MPCNL complications; and *P* value <0.05 was considered to be statistically significant.

## 3. Result

### 3.1. Comparison of the Incidence of Complications of CDCS in MPCNL

According to CDCS, totally there were 390 cases in MPCNL complications; the cases of grade I, II, III, IV, and V complications were 6.92% (27 cases), 8.21% (32 cases), 2.82% (11 cases), 1.79% (7 cases), and 0.26% (1 case), respectively. Among these complications, the proportion of cases with fever (body temperature ≧ 39°C) was the largest (4.87%), the complications within grade III were 70 cases (89.74%), mainly including urinary infections and blood transfusion caused by intraoperative bleeding, and the proportion of infection and blood transfusion was 4.10% and 3.08%, respectively; there was 1 patient who died of acute myocardial infarction. The results are shown in Table 1.

### 3.2. Comparison and Analysis of Clinical Data in Two Groups

There were no significant differences in gender, BMI, demographic characteristics, and anesthesia between the two groups (*P* > 0.05). Age (>60 years), associated comorbidities, preoperative albumin level (<35 g/L), stone complexity, operation time (>180 min), intraoperative bleeding volume (>300 ml), and hospital stays (>7 days) of the observation group (complication group) were significantly higher than that of the control group (noncomplication group). The results are shown in Table 2.

### 3.3. Multivariate Logistic Regression Analysis of Complications

78 patients with complications of MPCNL in perioperation were analyzed by multivariate logistic regression analysis, the results demonstrated that age (>60 years), associated comorbidities, preoperative albumin levels (<35 g/L), the stone complexity, the operation time (>180 min), and intraoperative bleeding volume (>300 ml) were associated with complications in patients by Claivien–Dindo classification. The results are shown in Table 3.

## 4. Discussion

Currently, MPCNL is one of the most common clinical treatments for renal stones. Percutaneous renal channel is F16 ∼ F20, which is far less than the traditional Fr 24 ∼ Fr 34. Thus, MPCNL can greatly shorten the area of the incision, reduce surgical injury, and increase the stone discharging rate. Some previous studies have reported that MPCNL promoted clinical efficacy, while some new complications appeared, which can lead to the increasing trend of total incidence rate of complications [13, 14]. CDCS began to be applied for clinical assessment of complications, with the improvement and update of CDCS in past decades, and surgical complications can be more detailed, reasonable, and objective to evaluate [15].

One researcher [16] analyzed the perioperative complications of 172 stone patients undergoing MPCNL using CDCS and showed that the overall incidence of complications was almost as high as 30%, with 9.88%, 6.98%, 7.56%, 3.49%, and 0.58% of class I, II, III, IV, and V complications, respectively. Nevertheless, the total incidence of complication of this study was 20.00% (78/390), and the incidence of complication of grade I, II, III, IV, and V were 6.92% (27/390), 8.21% (32/390), 2.82% (11/390), 1.79% (7/390), and 0.26% (1/390), respectively. The total incidence of complications and the complications of grade III and IV were reduced, and the possible explanations may be related to the differences of surgeons' experience and improvements in technology and equipments. Zeng et al. [17] adopted the CDCS to classify the perioperative complications of 377 patients in MPCNL, and the results showed that the associated comorbidities, stone complexity, and urinary abnormal anatomy were closely correlated with occurrence of perioperative complications. In this study, part of the results was similar as the results of Zeng et al [17]; moreover, our results agreed that the age, preoperative albumin levels, operation time, and intraoperative bleeding volume were the risk factors of perioperative complications of stones in patients.

In this study, the major complications in MPCNL were fever, infections, and bleeding within grade III of CDCS, which were the most common three adverse reactions, but grade IV∼V of CDCS were major threats to the life security of patients. Therefore, the analysis of factors related to the occurrence of complications of CDCS can provide reference data for the managements of preoperative assessment and surgical scheme. According to the results of multivariate logistic regression analysis, the possible reasons may be explained in terms of these risk factors. Firstly, patients with age >60 years were often complicated with one or more comorbidities, and this will result in the decrease of coagulation function, body organic function, and surgical tolerance [18, 19]. Secondly, albumin is the common protein in plasma, which can reflect the condition of liver function and body immunity at a certain extent [20], and once the liver function was impaired, albumin levels were also reduced; meanwhile, there were obstacles in coagulation function and body immunity. Thirdly, urinary abnormal anatomy, large size stones, and complex location stones will increase the difficulties of fragmenting and discharging of stones [21, 22]. Lastly, the longer operation time and wound exposure time will increase the risk of bacterial infections and the volume of bleeding, and these risk factors mentioned above were influenced each other and increased the probability of complications, and made an interactive effect to deteriorate the safety profiles on patients [23].

In this study, several viewpoints must be presented for prevention and management of complications in MPCNL. If severe skeletal deformities, urinary abnormal anatomy, or hydronephrosis were not obvious, puncture should be performed under the B ultrasonic or C-arm on necessity of avoiding the main blood vessels. Once the main renal blood vessels injured and large bleeding appeared, nephrostomy tube should be immediately closed, and immediate hemostasis must be taken [24, 25]. Referring to elderly patients with poor nutritional status or complicated with several comorbidities, the related examinations and preassessment should be well performed before operation [18]. In this study, one patient died of acute myocardial infarction, which reminded urologists that they must carry out more rigorous preoperative assessment for these elderly patients complicated with comorbidities.

In conclusion, the CDCS can give standard and more comparative criteria for the assessment of perioperative complications in MPCNL, and the urologists should pay more attention to these high-risk factors, which will provide reference data to ensure surgical safety and promote the clinical efficacy.

## Figures and Tables

**Table 1:** Comparison of CDCS of MPCNL complication in 390 patients (*n* (%)).

Grade	Complications	Incidence rate
Grade I		27 (6.92%)
	Body temperature ≧39°C	19 (4.87%)
	Increase of CCR, (alanine aminotransferase) ALT	5 (1.28%)
	Application of analgesic drugs	3 (0.77%)
Grade II		32 (8.21%)
	Blood transfusion caused by intraoperative bleeding	12 (3.08%)
	Urinary infections	16 (4.10%)
	Perirenal effusion	4 (1.03%)
Grade IIIa		8 (2.05%)
	Urinary tract obstruction	3 (0.77%)
	Closed drainage of thoracic cavity	2 (0.51%)
	Embolization of renal artery caused by bleeding	1 (0.26%)
	Renal pelvis perforation	1 (0.26%)
Grade IIIb		3 (0.77%)
	Renal abscess	2 (0.51%)
	Unilateral nephrectomy	1 (0.26%)
Grade IVa		6 (1.54%)
	Myocardial infarction	2 (0.51%)
	Cerebral stroke	2 (0.51%)
	Colonic injury	1 (0.26%)
	Acute renal failure	1 (0.26%)
Grade IVb		1 (0.26%)
	Shock	1 (0.26%)
Grade V		1 (0.26%)
	Death	1 (0.26%)

**Table 2:** Comparison of complications in two groups (*n* (%)).

Items		Observation group (78)	Control group (312)	*χ* ^2^	*P*
*Gender*					
	Male	52 (66.67%)	207 (66.35%)	0.052	0.820
	Female	26 (33.33%)	110 (33.65%)		
*Age (years)*					
	>60	59 (75.64%)	193 (61.86%)	5.184	0.023
	≦60	19 (24.36%)	119 (38.14%)		
*BMI (body mass index) (kg/m* ^*2*^)					
	>23	46 (58.97%)	190 (60.90%)	0.097	0.756
	≦23	32 (41.03%)	122 (39.10%)		
*Demographic characteristics*					
	Urban	55 (70.51%)	219 (70.19%)	0.003	0.956
	Rural	23 (29.49%)	93 (29.81%)		
*Associated comorbidities*					
	Yes	30 (38.46%)	136 (24.36%)	6.270	0.012
	No	48 (61.54%)	176 (75.64%)		
*Preoperative albumin (g/L)*					
	≧35	65 (83.33%)	217 (69.55%)	6.843	0.009
	<35	12 (16.67%)	95 (30.45%)		
*Stone complexity*					
	Simple	39 (50.00%)	216 (69.23%)	10.196	0.001
	Complex	39 (50.00%)	96 (30.77%)		
*Operation time (min)*					
	>180	55 (70.51%)	96 (30.76%)	41.541	≤0.001
	≦180	23 (29.49%)	216 (69.23%)		
*Intraoperative bleeding volume (mL)*					
	>300	42 (53.85%)	114 (36.54%)	8.337	0.004
	≦300	35 (46.15%)	198 (63.46%)		
*Hospital stays (d)*					
	>7	47 (60.26%)	135 (43.27%)	7.235	0.007
	≦7	31 (39.74%)	177 (56.73%)		
*Anesthesia methods*					
	Epidural anesthesia	54 (69.23%)	201 (64.42%)	0.637	0.425
	General anesthesia	24 (30.77%)	111 (35.58%)		

**Table 3:** Results of multivariate logistic regression analysis of Clavien–Dindo classification of complications in perioperation.

Items	B	Sb	Wald	*P*	OR	95%CI
Age	1.082	0.075	205.618	≤0.001	1.142	0.985–3.420
Associated comorbidities	0.983	0.185	28.264	≤0.001	1.125	0.783–3.8404
Preoperative albumin levels	2.465	0.317	60.279	≤0.001	4.412	2.398–21.917
Stone complexity	2.146	0.224	92.159	≤0.001	3.126	2.017–13.252
Operation time	1.017	0.126	65.052	0.003	2.562	2.001–3.540
Intraoperative bleeding volume	2.016	0.220	83.936	≤0.001	3.765	2.446–11.557

## Data Availability

The simulation experiment data used to support the findings of this study are available from the corresponding author upon request.
